The article "Effect of Foot and Hand Massage on Abdominal Pain of Cesarean Section Incision under Ultrasound Guidance" was retracted in 2023. Reasons: signs of a paper mill; suspected computer-generated content; unreliable results or conclusions; lack of ethics approval or compliance.

# Effect of Foot and Hand Massage on Abdominal Pain of Cesarean Section Incision under Ultrasound Guidance

**DOI:** 10.1155/2022/8356256

**Published:** 2022-07-27

**Authors:** Yu Qing Wang, Rongrong Jiang, Jianmin Pan

**Affiliations:** ^1^Pregnant Women School, Changyi People's Hospital, Weifang, Shandong 261300, China; ^2^Delivery Room, Changyi People's Hospital, Weifang, Shandong 261300, China

## Abstract

In order to relieve the pain of incision after cesarean section, a method of foot and hand massage for abdominal pain of cesarean section incision under ultrasound guidance was proposed in this paper. In this paper, the experimental control method and retrospective analysis were used to relax the patients through massage, so that the pregnant women could focus on the reaction caused by hand and foot massage, distract their attention, and reduce the pain. The results showed that 60 cases of puerpera after cesarean section were divided into two groups with 30 cases in each group. The control group was only given routine care. The intervention group received 20 min hand and foot massage on the basis of routine care. The visual analog scale (VAS) of pain before, immediately after, 30 min after, and 60 min after massage in the intervention group was evaluated and recorded, and the VAS scores of the control group at the corresponding time points were recorded. The VAS score of the intervention group at each time point after massage was significantly lower than that before massage (*P* < 0.05), and the VAS score of the intervention group at each time point was significantly lower than that of the control group (*P* < 0.01). Hand and foot massage can effectively relieve incision pain after cesarean section.

## 1. Introduction

Pregnancy and childbirth are normal physiological processes of human reproduction. Most women can naturally give birth to healthy babies. Cesarean section refers to the obstetric operation to remove the fetus and its appendages by cutting the abdominal wall and uterine wall after 28 weeks of pregnancy. Cesarean section is an important means to solve dystocia and some high-risk pregnancies and save the lives of mothers and infants.

With the development of society, cesarean section has become one of the important ways for parturients to deliver. It is an important means to solve many obstetric conditions, such as cephalopelvic disproportion, fetal malposition, and fetal distress, and reduce the maternal and neonatal mortality [1]. As well as the improvement of pregnant women's requirements for delivery, the cesarean section rate remains at a high level. In the number of deliveries, 1593425 cases had cesarean section, and the cesarean section rate was 50.67%. From 2019 to 2021, the age standardized cesarean section rates were 52.37%, 49.90%, 49.75%, 51.13%, and 50.66%, respectively, showing a downward trend first and then an upward trend (Figure 1). The average age of cesarean section delivery was 28.23 years, and the average age of noncesarean section delivery was 26.49 years.

It is necessary to further clarify the relevant factors that affect the choice of cesarean section for pregnant women, so as to provide corresponding basic support for this study. The analysis results of this study show that the independent factors affecting cesarean section include age, education level, registered residence, type of delivery hospital, prepregnancy BMI, maternal type, mode of pregnancy, adverse pregnancy and childbirth history, pregnancy complications or complications, and the number of pregnancy examinations. The cesarean section rate of pregnant women in area B is still high, as shown in Table 1.

After cesarean section, the anesthetic effect gradually subsides, and the pain sensation of lower abdominal incision begins to recover. Generally, it is most obvious within 24 h after the operation, which not only brings discomfort to the body but also psychological damage [2]. Pain is defined as the fifth vital sign after the four vital signs of body temperature, pulse, respiration, and blood pressure [3]. Therefore, relieving the incision pain after cesarean section has become one of the important tasks of nursing staff [4]. Pain after cesarean section is an important factor affecting the postoperative recovery and lactation of parturients. Good analgesia can reduce pain response and promote rapid postoperative recovery and postoperative lactation. The traditional methods of clinical analgesia are mainly epidural analgesia and intravenous analgesia. The effect of epidural analgesia is good, but it needs to retain epidural catheter (Figure 2). It is difficult to manage after operation. Maternal activities are easy to lead to catheter prolapse, motor block, urinary retention, and other adverse reactions. Intravenous analgesia is easy to use and manage, but opioid analgesics are prone to respiratory depression, excessive sedation, nausea, vomiting, and other adverse reactions. Multimodal analgesia is increasingly used in clinic to improve the analgesic effect and reduce adverse reactions. However, at present, there are still deficiencies in pain control after routine analgesia [5]. Ultrasound-guided foot and hand massage is effective in relieving postoperative incision pain [6]. The purpose of this study is to explore the intervention effect of foot and hand massage guided by ultrasound on incision pain of patients after cesarean section, to seek intervention methods to relieve their pain to the greatest extent, and to provide scientific basis for clinical practice [7].

## 2. Literature Review

There are many reasons for the postoperative pain of parturients. The most important ones are the pain of incision and the uterine contraction pain caused by the recovery of uterus, and the uterine contraction pain is more obvious after operation. With the disappearance of anesthetics after cesarean section, pregnant women will feel pain. The pain is not only limited to incision pain but also accompanied by contractile pain caused by intravenous oxytocin. If postoperative analgesia is not used, the degree of pain is mostly severe (VAS > 7 points) [8]. It can be seen from Table 2 that compared with cesarean section, the estimated value, real value, and recall value of pain in natural delivery were slightly higher, but the difference was not statistically significant (*P* > 0.05). There was no significant difference in the predicted value, the true value, and the recall value of pain among the parturients who gave birth naturally (*P* > 0.05). The estimated value of pain in cesarean section women was significantly lower than the real value, and the difference was statistically significant (*P* < 0.05). It can be seen from Table 3 that the estimated pain value of the parturients who choose cesarean section actively or passively is far lower than the real value, and the difference is statistically significant (*P* < 0.05).

The expectation of cesarean section women on delivery pain is far lower than the real experience value, while the estimated pain value of active cesarean section women is lower than the real value, indicating that the expectation of active cesarean section women on reducing production pain through surgical delivery is too high. Especially for the parturients who strongly expressed that they could not bear the pain of natural delivery and chose cesarean section, even after giving postoperative analgesia, they still had a deeper memory of the pain during delivery than the parturients who gave birth naturally. However, the estimated value of pain during delivery of the women who passively choose cesarean section is higher than the postpartum recall value. The reason for analysis may be that the women have a certain understanding of cesarean section and postoperative pain, so that they have a better psychological preparation. On the other hand, it is related to the fact that they pay more attention to the safety of mother and baby than to the pain.

In the past, continuous patient-controlled epidural analgesia and patient-controlled intravenous analgesia were used [9]. Patient controlled epidural analgesia (PCEA) has a definite effect, but it has some disadvantages, such as urinary retention, numbness of both lower limbs, inability to get out of bed early, and easy to fall off of epidural catheter due to turning over, which affect its clinical application. In the simple patient-controlled intravenous analgesia mode, individual sensitivity to drugs may easily lead to large individual differences in medication effects. Some people use large amounts of drugs, and the incidence of adverse reactions such as dizziness, nausea, and vomiting is high [10].

Massage can promote qi and blood circulation, dredge meridians, and achieve the purpose of pain relief [11]. Moreover, pain receptors are generally located in the skin and subcutaneous tissue, and the most dense places are the hands and feet. After mechanical stimulation, the receptors on the body surface are transmitted to the brain along the spinal cord, and then, the brain sends information to excite the vagus nerve to act on the hypothalamus, which promotes the increase of enkephalin and dynorphin, the content of pain causing substances in the body, and affects the secretion and metabolism of pain-related neurotransmitters, hormones, and the evolution and release of chemical substances in the body, thus playing the role of analgesia. Therefore, the use of hand and foot joint massage to relieve postoperative pain is a valuable intervention [12].

## 3. Method

### 3.1. Object Selection

60 cases of cesarean section in hospital B were selected as data samples, of which the main age was 18-40 years (27.3 ± 4.8 years). They were randomly divided into control group and intervention group, with 30 cases in each group. Inclusion criteria are as follows: those with normal cognition; volunteer to participate in the study; it conforms to grades I and II of the American Society of Anesthesiologists' disease classification standard; and those who have undergone cesarean section [13]. Exclusion criteria are as follows: patients with consciousness disorder and psychosis; postoperative patient-controlled analgesia; damaged tissue and skin of hand or foot, phlebitis, arthritis, burn wound, inflammation, eczema, etc.; and pregnant women with heart disease, high blood pressure, and excessive intraoperative bleeding. There was no significant difference between the two groups in educational level, age, place of residence, gestational weeks, and anesthesia methods (*P* > 0.05).

### 3.2. Massage Method

#### 3.2.1. Intervention Methods

This study adopts the clinical trial research method [14]. The control group was given routine nursing, and the intervention group was given 20 min hand and foot massage on the basis of routine nursing. On the first day before operation, explain the use of visual analogue scale (VAS) for pain to the pregnant women who volunteered to participate in the study. On the first day after operation, provide a comfortable place for pregnant women. The room temperature is controlled at 18°C~22°C, keep the environment quiet, and the bed is clean, dry, and free of debris [15]. Before intervention, the operator washed his hands, cut his nails, did not wear jewelry, rubbed his hands to keep them warm, and asked the patient to lie flat. On the basis of consulting relevant experts and consulting literatures, the massage steps were formulated: put the thumbs of both hands in the middle of the back of the patient's hands and the other four fingers close to the palm of the hand to do the action of grasping and sliding. Turn the patient's hand over, place the two thumbs of the operator in the middle of the patient's palm, and stick the other four fingers on the back of the hand. The two thumbs slide from the center of the hand to the left and right sides and then return to the origin, so as to massage the thenar, 2 or 3 times for each hand. After the hand massage, one hand holds the foot, the other half clenches the fist, the index finger bends, and apply force to the vertex of the first finger joint of the index finger. During the pressing, keep the index finger bones in line with the palm, forearm, and big arm, and the force should be appropriate and uniform. According to the patient's sensitivity to pain, grasp the massage force properly, press the corresponding part of the foot reflection area as a whole, and then fix the patient's foot and ankle, with the palm facing the patient's foot bottom, help them flex and extend their toes for 10~15 times, and do the opposite side with the same method.

#### 3.2.2. Measuring Tools

In this study, general information questionnaire and VAS were used as data collection tools. Measure and record the pain intensity of the intervention group before massage, immediately after massage, 30 min after massage, and 60 min after massage, and record the pain of the control group at the corresponding time point [16]. The general information questionnaire is designed by the researcher according to the research needs and perfected under the guidance of relevant experts, including age, occupation, education level, and residence. VAS is to draw a straight line on the paper, with 0 and 10 marked on both ends, respectively. 0 represents no pain, and 10 represents the most severe pain. Let the puerpera mark the number on the straight line according to the degree of incision pain they feel; that is, score the pain intensity of the puerpera. VAS is an effective tool commonly used in scientific research and clinical practice. Its reliability and validity in pain assessment have been proved.

#### 3.2.3. Statistical Methods

Medical statistics is an important tool for medical research. It is widely used in experimental design, data collection, and data analysis. The correct application of statistical methods has an extremely important significance and role in effectively carrying out scientific research and improving the academic quality of medical scientific papers. The basic methods of statistics are generally not difficult to master, but whether they can be correctly used is still a common problem.

SPSS19.0 software will be used for statistical analysis of the data in this paper. The main statistical methods include *t*-test and repeated measurement analysis of variance [17].

*(1) Repeated Measurement Method*. Repeated measurement method is widely used in medical research, such as clinical research on the short-term and long-term efficacy of a certain treatment method, blood drug concentration of different doses of the same drug at various time points after use, etc. The repeated measurement design is used to analyze the change trend of observation indicators and related influencing factors, and the repeated measurement data are arranged in time. The randomized block design is mainly to control the influence of other factors other than the treatment factors on the test results, so that the treatment groups can be balanced and comparable as far as possible. Therefore, the data between the treatment groups are independent. According to the output results of SPSS19.0, we can sort out the results as shown in Table 4.

*(2) *t*-Test*. *t*-test is a hypothesis test method established by the British statistician W.S. Gosset based on the *t*-distribution principle in 1908. It is often used to compare the mean of two small samples in the measurement data. In theory, the application condition of *t*-test is that the sample is from the population with normal distribution. When comparing the mean of two samples, it also requires that the variance of the two populations be equal. However, in practice, it deviates slightly from the above conditions. As long as its distribution is unimodal and approximate normal distribution, it can also be applied.

There are three types of *t*-tests commonly used: (1) *t*-test of single sample: it is used to infer whether the population mean represented by the sample mean and the known population mean has statistical significance. When the number of samples is small (*n* < 60) and the overall standard deviation is unknown, *t*-test is used. On the contrary, when the number of samples is large or small, and the overall standard deviation is known, *U*-test can be used. (2) Paired specimen *t*-test: it is applicable to the comparison of the mean number of two specimens in the paired design. When selecting, attention should be paid to whether the two specimens are paired design data. The commonly used paired design data mainly include the following three cases: two homogeneous subjects receive two different treatments, respectively. The same subject or two parts of the same specimen were treated differently. Compare the results of the same subject before and after treatment. (3) *t*-test of two independent samples: also known as group *t*-test, it is applicable to the comparison of the mean of two samples with completely random design. Different from the paired *t*-test, before the *t*-test of two independent samples, the homogeneity of variance test must be carried out for the two groups of data. If it is a small sample with homogeneous variance, *t*-test is used. On the contrary, if the variance is not uniform, the corrected *t*-test (t-test) is used, or the data transformation method (such as logarithm, square root, and reciprocal) is used to make the two groups of data have the homogeneity of variance before the *t*-test, or the nonparametric test is used. In addition, when the number of samples in the two groups is large (*N*1, *n*2 > 50), the calculation of *t*-test is cumbersome, and *U*-test can be used.

## 4. Results and Discussion

### 4.1. Result Analysis

There was significant difference in VAS scores at each time point in the intervention group (*P* < 0.01). There were significant differences in VAS scores between two groups at different time points in the intervention group (*P* < 0.05). There was no significant difference in VAS score of the control group at each time point (*P* > 0.05). The VAS scores of the intervention group at each time point after massage were significantly lower than those of the control group (*P* < 0.01) (see Table 5).

### 4.2. Result Discussion

#### 4.2.1. Role of Hand and Foot Massage

The results of this study show that after the analgesic effect of anesthetics disappears after cesarean section, routine nursing has no significant effect on postoperative incision pain of parturients [18]. However, the VAS at 30 min after massage intervention was the lowest (2.67 ± 0.71), which was significantly lower than that before massage. Although the VAS at 60 min after massage rose again, it was still lower than that before massage [19]. The comparison between the two groups showed that the VAS score of the intervention group after massage was lower than that of the control group, suggesting that hand and foot massage can reduce the intensity of incision pain of pregnant women after cesarean section. The results of this study are similar to those of foreign scholars. The joint massage of hands and feet for 20 min can effectively relieve the postoperative pain of dissecting uterus parturients, and the effect of massage lasted until 60 min after massage, and the degree of pain increased slightly 90 min after massage.

#### 4.2.2. Principle of Hand and Foot Massage for Relieving Incision Pain after Cesarean Section

Massage is a natural health care method that integrates the meridian theory, modern pathophysiology, bioholographic embryo theory, reflection theory, etc. [20]. Traditional Chinese medicine believes that “if there is no obstruction, there will be pain, and if there is general, there will be no pain.” After the operation, the blood of the meridians overflows outside the veins and remains in the skin, resulting in qi stagnation and blood stasis, and blocked channels. Massage can promote qi and blood circulation, dredge meridians, and achieve the purpose of pain relief. Moreover, pain receptors are generally located in the skin and subcutaneous tissue, and the most dense places are the hands and feet [21]. The receptors on the body surface are mechanically stimulated and transmitted to the brain along the spinal cord, and then, the brain sends information to excite the vagus nerve to act on the hypothalamus, which promotes the increase of enkephalins and dynorphins and the decrease of the content of pain causing substances in the body. It affects the secretion and metabolism of neurotransmitters and hormones related to pain and the evolution and release of chemicals in the body, thus playing an analgesic role. In addition, massage brings relaxation to the patient, which makes the pregnant woman focus on the reaction caused by hand and foot massage, distracting her attention, thus reducing the pain.

## 5. Conclusion

This paper presents a method of foot and hand massage for abdominal pain in cesarean section incision under ultrasound guidance. Massage can promote qi and blood circulation, dredge meridians, and achieve the purpose of pain relief. Pain receptors are generally located in the skin and subcutaneous tissue, and the most dense places are the hands and feet. The receptors on the body surface are mechanically stimulated and transmitted to the brain along the spinal cord, and then, the brain sends information to excite the vagus nerve to act on the hypothalamus, which promotes the increase of enkephalin and dynorphin and the decrease of the content of pain causing substances in the body. It affects the secretion and metabolism of neurotransmitters and hormones related to pain and the evolution and release of chemicals in the body, thus playing an analgesic role. In addition, massage brings relaxation to the patient, which makes the pregnant woman focus on the reaction caused by hand and foot massage, distracting her attention, thus reducing the pain. In the high-cost medical care environment, using hand and foot joint massage to relieve postoperative pain is a valuable intervention, which improves the nursing level of nurses for postoperative pain.

## Figures and Tables

**Figure 1:** Time trend of cesarean section rate from 2019 to 2021.

**Figure 2:** Cesarean section incision.

**Table 1:** Results of multifactor analysis on influencing factors of cesarean section among parturients in area B.

Influence factor	Classification	*β*	SE	Wald *χ*^2^ value	*P* value	OR (95% CI)
Age (years)	20 ~ 24 = 1, 25 ~ 34 = 2, and >35 = 3	1.456	0.612	5.660	0.017	4.289 (1.292~1.4232)
Degree of education	Junior high school and below = 1, high school = 2, and college degree or above = 3	0.451	0.101	19.939	<0.001	1.570 (1.288~1.914)
Registered residence (rural as reference)	City	0.734	0.277	7.022	0.008	2.083 (1211~3.586)
Type of delivery hospital (township/town level as reference)	District/county level	0.342	0.215	2.530	0.065	1.408 (0.924~2.146)
	Municipal level and above	1.158	0.329	12.389	<0.001	3.184 (1.677~6.067)
Prepregnancy BMI (kg/m^2^, 18.5~23.9 as reference)	<18.5	0.734	0.465	2.492	0.065	2.083 (0.837~5.183)
	24.0~	0.158	0.219	0.521	0.853	1.171 (0.762~1.799)
	>28.0	0.685	0.165	17.235	<0.001	1.984 (1.436~2.741)
Maternal type (primipara as reference)	Parturient women	-1.347	0.224	36.161	<0.001	0.260 (0.168~0.403)
Fertility formula (multiple photos for natural pregnancy)	Assisted reproduction	0.403	0.078	26.694	<0.001	1.496 (1.284~1.743)
Adverse pregnancy and childbirth history (no as reference)	Yes	0.902	0.450	4.018	0.045	2.465 (1.020~5.954)
Complications or complications during pregnancy (no as reference)	Yes	2.426	0.545	19.815	<0.001	11.314 (3.888~32.924)
Times of antenatal examination (<5 as reference)	5~7	0.333	0.171	3.792	0.052	1.395 (0.998~1.951)
	≥8	0.790	0.379	4.345	0.047	2.203 (1.048~4.631)

**Table 2:** Comparison of maternal pain scores in different delivery modes ($\bar{x}$±s, points).

Mode of delivery	Estimated value	True value	Recall value	*F*	*P*
Spontaneous childbirth	3.80 ± 0.84	4.63 ± 0.554	4.42 ± 0.894	1.444	0.274
Cesarean section	3.01 ± 0.71	4.60 ± 0.54a	4.04 ± 0.960	5.442	0.021
*t*	1.372	-0.343	1.177		
*P*	0.242	0.749	0.305		

a: estimated value comparison, *P* < 0.05.

**Table 3:** Comparison of pain scores of cesarean section women with different selection methods ($\bar{x}$±s, points).

Selection method	Estimated value	True value	Recall value	*F*	*P*
Active selection	2.86 ± 0.44	4.40 ± 0.53^a^	3.82 ± 0.84	5.360	0.022
Passive selection	3.44 ± 1.14	4.80 ± 0.45^a^	3.03 ± 0.97	8.167	0.006
*t*	0.885	1.002	−2.138		
*P*	0.426	0.374	0.099		

a: estimated value comparison, *P* < 0.05.

**Table 4:** Repeated measurement ANOVA results.

Source of variation	Sum of squares of deviation from mean	Freedom	Mean square	*F*	*P*
Treatment factors	23.361	1	23.361	79.340	<0.001
Time factor	24.389	2	12.194	30.276	<0.001
Processing factor ∗ time factor	17.056	2	8.528	21.172	<0.001
Individual error	2.944	10	0.294		
Repeated measurement error	8.056	20	0.403		

**Table 5:** Comparison of VAS scores of the two groups at different time points ($\bar{x}$±s).

Group	Number of cases	Before massage	Immediately after massage	30 min after massage	60 min after massage	*F* value	*P*
Control group	30	5.50 ± 0.57	5.63 ± 0.72	5.93 ± 0.74	5.70 ± 0.70	2.301	>0.05
Intervention group	30	5.53 ± 0.86	3.10 ± 0.80^1)^	2.67 ± 0.71^1)2)^	3.60 ± 1.00^1)2)3)^	110.220	<0.01
*t* value		-0.18	12.88	17.437	9.391		
*P*		>0.05	<0.01	<0.01	<0.01		

1): compared with before massage, *P* < 0.05; 2): compared with immediately after massage, *P* < 0.05; 3): compared with 30 min after massage, *P* < 0.05.

## Data Availability

The data used to support the findings of this study are available from the corresponding author upon request.
